The article "Identifying the Impact of Industrial Agglomeration on China's Carbon Emissions Based on the Spatial Econometric Analysis" was published in 2023. Journal: J Environ Public Health.

# Identifying the Impact of Industrial Agglomeration on China's Carbon Emissions Based on the Spatial Econometric Analysis

**DOI:** 10.1155/2023/4354068

**Published:** 2023-01-31

**Authors:** Xianpu Xu

**Affiliations:** School of Business, Xiangtan University, Xiangtan 411105, China

## Abstract

China's rapid economic growth is accompanied by industrial agglomeration (IA) and environmental pollution. Although IA has played an important role in reducing environmental pollution, its effect on carbon emissions is still debatable and deserves further study. In this context, this paper constructs a two-sector general equilibrium model including households and firms to explore the mechanisms of IA on carbon emissions and finds that IA mainly affects carbon emissions through the agglomeration effect and congestion effect. Then, based on the balanced panel data for 30 Chinese provinces from 2003 to 2019, this study employs the dynamic spatial panel model to investigate the nexus between different types of IA and carbon emissions. The empirical results reveal that a significant positive spatial dependence is verified in the regional carbon emissions of China, indicating that carbon emissions exhibit a remarkably spatial spillover effect. Meanwhile, there are significant variations in the influence of different types of IA on carbon emissions. Specifically, specialized agglomeration (SA) positively affects carbon emissions, while the impact of diversified agglomeration (DA) on carbon emissions is negative, implying that China's DA may contribute to carbon emission control. In addition, there is regional heterogeneity in the effect of IA on carbon emissions, with the western region having a significantly greater effect than the eastern and central regions. Therefore, the Chinese government should follow the notion of integrating territory administration and interregional communication and formulate regionally differentiated environmental governance policies to promote carbon emission reduction in the future.

## 1. Introduction

Climate change, which is mainly characterized by global warming, has seriously endangered the living environment of human beings and it is recognized as one of the most challenging problems facing mankind today [1]. Reducing carbon emissions and promoting low-carbon development have become the critical tasks around the world [2]. Since the reform and opening up in 1978, China has achieved a remarkable growth miracle, which was mainly driven by industrialization. According to the data released by the National Bureau of Statistics in 2018, the average annual growth rate of China's gross domestic product (GDP) is up to 9.5% over the period 1980–2015. However, the extensive economic growth has brought about massive carbon emissions due to the features of high energy consumption, high pollution, and low output, as shown in Figure 1. In 2007, China became the global largest carbon emitter, which has severely affected the development of China's regional economy in a sustainable manner [4]. Due to the global push to reduce carbon emissions and huge pressure from the carrying capacity of domestic resources and environment, China's efforts to reduce carbon emissions have become the focus of the international community. As a responsible developing country, China has taken positive actions in climate governance and proposed a series of binding targets for emission reduction. Specifically, at the Copenhagen Climate Summit in late 2009, China pledged to cut carbon emissions per unit of GDP by 40%–45% by 2020 compared to 2005. Moreover, according to the 2015 Paris Agreement, China also stated that it will cut its carbon emissions per unit of GDP by 60%–65% and add forest stock volume by 4.5 billion cubic meters by 2030 compared to the 2005 levels. In 2020, China announced that carbon emissions would peak around 2030 and achieve carbon neutrality by 2060, demonstrating China's commitment to realizing its carbon-reduction targets. In order to realize the green and sustainable development in China, it is necessary to optimize the energy consumption structure and enhance carbon productivity instead of simply relying on increasing factor inputs. Under such circumstances, what is the effect of China's carbon emissions reduction? What kind of reduction paths should be established to achieve the goal of “carbon peak and carbon neutrality”? Answering these questions has an important significance for improving the quality of the ecological environment and promoting the high-quality development of China's economy [5].

The article "Identifying the Impact of Industrial Agglomeration on China's Carbon Emissions Based on the Spatial Econometric Analysis" was published in 2023. Journal: J Environ Public Health.

In the process of economic development, production factors and economic activities are relatively concentrated in a certain geographical space, which was be known as IA [6, 7]. In recent years, the Chinese government has developed a range of positive and upgrading industrial policies to promote economic growth. For example, in order to achieve industrialization by 2025 and become a manufacturing power, the State Council issued a document named “Made in China 2025” in 2015, which is a strategic document to promote the implementation of manufacturing power comprehensively. Meanwhile, the 13th Five-Year Plan, which includes the National Strategic Emerging Industry Development Plan, was also released by the State Council in 2016, which requires accelerating the growth of strategic emerging industries and vigorously building a new modern industrial system. In addition, the Fifth Plenary Session of the 19th Central Committee of CPC advocated a plan that accelerated the development of a modern industrial system and promoted the modernization of the industrial chain. The continuous development of the industry is accompanied by IA. Theoretically, as an important mode of economic development and an inevitable trend of industrial development, IA and economic growth are mutually reinforcing. Specifically, IA can significantly optimize the allocation of input factors and improve the production efficiency of enterprises, which can contribute to economic growth [8]. However, in the later stages of agglomeration economy development, there are some negative externalities caused by excessive competition and congestion effects in the agglomeration areas, which intensifies energy consumption and overcapacity [9]. In addition, with China's economic growth having moderated to a “new normal” pace, the quality of economic development should be highly considered now. In this context, is it possible for China's IA to attain a win-win scenario in terms of both economic growth and environmental protection? In other words, can China's IA help reduce environmental pollution, especially carbon emissions caused by reliance on fossil energy? Will the impact of IA on carbon emissions change due to the form of agglomeration? In addition, owing to the huge regional disparities in China, the degree of industrialization varies across different regions. Then, is there regional heterogeneity in the effect of IA on carbon emissions? Obviously, exploring these issues has a very important significance for clarifying the factors influencing China's carbon emissions and formulating differentiated industrial policies to promote carbon emission reduction.

The purpose of this study is to explore the nexus between different forms of IA and China's carbon emissions from the perspective of spatial spillover. Specifically, by constructing a two-sector growth model, we first analyze the influence mechanisms of IA, which is divided into SA and DA, on carbon emissions. Then, by using a panel data for China's 30 provinces during 2003–2019, we calculate the level of carbon emissions for each province and employ Moran's I test to investigate the spatiotemporal evolutionary characteristics of China's regional carbon emissions. Furthermore, the spatial dynamic panel econometric model is used in this paper to explore the relationship between IA and carbon emissions. Considering the regional heterogeneity, we conduct regional heterogeneity analysis to verify the heterogeneous effects in different regions. Our main findings are listed below. First, there is a significant positive cumulative effect and spatial lag effect, as well as a negative spatiotemporal lag effect in China's carbon emissions, which indicates that the amount of carbon dioxide emitted in the region will be affected by adjacent regions. Second, different forms of IA have significantly different impacts on carbon emissions. Specifically, SA promotes carbon emissions, while DA inhibits carbon emissions. Third, the impacts of urbanization and infrastructure on carbon emissions are both significantly negative, but the impact of economic development is not significant. Meanwhile, there is an inverted U-shaped nexus between carbon emission and environmental regulation. Finally, at the regional level, the impact of IA on carbon emissions varies considerably, with the western region having a greater effect than the eastern and central regions.

The article "Identifying the Impact of Industrial Agglomeration on China's Carbon Emissions Based on the Spatial Econometric Analysis" was published in 2023. Journal: J Environ Public Health.

The main contributions of this paper to the existing literature can be outlined below. First, based on an endogenous growth model, the transmission mechanisms of IA on carbon emission are deeply analyzed in this study. Specifically, by incorporating IA and carbon emission into a unified analytical framework, we provide new insights for the causes of carbon emissions and the governance mode of environmental pollution in China, which contributes to give full play to the industrial advantages of different regions and promote green development of China's economy. Second, in order to illustrate whether the different mode of IA can improve China's carbon emissions, IA is divided into SA and DA, and the influence of IA on carbon emissions is then comprehensively investigated from the two dimensions, which expands the research perspective and makes up for the shortcomings of the existing literature. In addition, explaining how to reduce carbon emissions from the perspective of the mode of IA can provide useful decision-making references for optimizing China's regional industrial structure, promoting the rational layout of IA, and realizing the sustainable development of China's economy. Finally, we use the dynamic spatial lag model to analyze the nexus between IA and carbon emissions based on provincial panel data in China over the period from 2003 to 2019. The majority of existing studies on carbon emissions were based on non-spatial empirical methods, which fails to explain the conclusions of research effectively. However, the effects of IA on carbon emissions may be revealed in a more reasonable and accurate manner due to the spatial econometric models paying more attention to the spatial spillover effects of carbon emissions in neighboring economies. Furthermore, the impact of IA on carbon emissions is explored from a spatial dependence perspective, which provides useful policy guidance for establishing an interregional joint prevention and control mechanism for China's carbon emission reduction and improving the level of environmental governance in different regions.

The article "Identifying the Impact of Industrial Agglomeration on China's Carbon Emissions Based on the Spatial Econometric Analysis" was published in 2023. Journal: J Environ Public Health.

The rest of this study is organized as follows.  Section 2 reviews the relevant literature.  Section 3 creates an endogenous growth model to explore the nexus between IA and carbon emissions.  Section 4 describes the data sources, variables, and econometric models.  Section 5 reports and analyzes the empirical estimation results.  Section 6 concludes the study and proposes several policy implications.

## 2. Literature Review

Through sorting out the prior research, the literature related to the study can be divided into three streams: IA and economic development, the influencing factors of carbon emissions, IA and carbon emissions. An overview of recent research relating to these topics is presented as follows.

The first stream examines the connection between IA and economic development. IA is defined as a process in which linked sectors are highly concentrated in a geographic region and capital elements are constantly converging [10]. Despite extensive research into the relationship between IA and economic growth, no consensus has been found. The mainstream view is that IA can help promote economic development. The agglomeration effect of IA, such as the scale effect and technology spillovers, can promote technological progress and improve factor productivity [11]. In addition, the shortening of the spatial distance reduces the information cost and transportation cost for firms, thereby improving economic development. This conclusion has been confirmed in several countries. Fan and Scott [12] discovered a positive nexus between IA and the economic growth of East Asian economies and confirmed that manufacturing agglomeration and labor productivity are highly correlated. Brülhart and Mathys [13] examined the linkage between IA and economic development by using a dynamic panel GMM and presented that IA can promote labor productivity in EU countries, thereby promoting economic growth. Similar conclusions were drawn by Liang and Goetz [14]. Conversely, some scholars hold the view that IA will inhibit economic growth. The excessive clustering of production factors in a region will inevitably accelerate the competition of enterprises in the factor market, cause vicious competition among enterprises, and lead to an increase in the price of factor resources, resulting in a congestion effect and hindering regional economic growth [15]. For example, Paci and Usai [16] demonstrated a weak negative correlation between technological concentration and total productivity for 109 regions in the European Union. Furthermore, a few studies show that a nonlinear linkage exists between IA and economic development because the positive and negative externalities of IA exist simultaneously and whether the agglomeration effect or the congestion effect appears depends on which effect ultimately dominates. Based on the sample data from 1996 to 2003 in Europe, Antonelli et al. [17] analyzed the impacts of economic agglomeration on the growth in regional productivity and verified that agglomeration and economic development follow an inverted U-shaped curve. Similar findings were obtained based on samples from the United States [18]. In conclusion, although existing literature has deeply analyzed the linkage between IA and economic development, the nexus between IA and carbon emissions has not aroused enough attention. Under the “Dual Carbon Goals,” how to balance economic development and the environment in IA is still a significant and urgent issue that must be addressed.

The article "Identifying the Impact of Industrial Agglomeration on China's Carbon Emissions Based on the Spatial Econometric Analysis" was published in 2023. Journal: J Environ Public Health.

The second stream related to this paper investigates the influencing factors of carbon emissions with the increasing attention to environmental issues [19–21]. Specifically, relevant literature can be classified into three parts according to driving factors, including the institutional level, the market level, and the economic environment level. From the perspective of institutional factors, the continuous improvement of the system speeds up the rational allocation of resources and reduces carbon emissions. For example, Mayor and Tol [22] argued that a carbon tax is an economic tool for reducing carbon emissions and preventing global climate change, and these findings were echoed by Wang et al. [23]. Bartle [24] believed that environmental policies and regulations can effectively control greenhouse gas emissions, and analyzed the theoretical mechanism between the two. Based on the OLS approach, Jiang and Ma [25] investigated and determined a U-shaped link between carbon emissions and environmental regulation. In addition, by using the panel data for 17 European Union countries during 1995–2017, Neves et al. [26] confirmed that market-based regulatory policies can reduce carbon emissions in the long-run. The conclusion was further verified by Croci et al. [27]. From the perspective of market factors, a fully functional market system is conducive to improving the price formation mechanism, standardizing the order of the carbon trading market, and curbing carbon emissions. Based on the panel data from a sample of 116 countries and the System-GMM estimation, Acheampong [28] examined the influence of energy consumption on carbon emissions and revealed that the consumption of energy promotes carbon emissions in the Middle East and North Africa. By using a dynamic threshold panel model, Wu et al. [29] investigated the nexus between environmental regulation, energy consumption, and carbon emissions. The findings indicated that increased energy consumption plays a key role in exacerbating carbon emissions, but this role has declined as environmental control has improved. Zhang et al. [2] studied the effects of energy taxes, energy prices, and population on carbon emissions in European countries and found that rising energy prices and energy taxes would reduce greenhouse gas emissions. Furthermore, it was discovered that carbon emissions increase as the population grew and decrease as the level of urbanization increases. From the perspective of economic environmental factors, there is no agreement on the link between carbon emissions and the economic environment. Pao and Tsai [30] concluded that there is an EKC hypothesis for three of the BRIC countries. As real output increases, carbon emissions first keep increasing, then tend to stabilize and finally decline. By using the data of 27 European Union countries from 1988 to 2009, Lee and Brahmasrene [31] explored the influence of tourism and economic growth on carbon emissions and found that tourism has a significant negative impact on carbon emissions, while economic growth is not. Umar et al. [20] used Chinese provincial panel data to analyze the drivers of carbon emissions, including economic growth, financial development, globalization, and natural resources. The results showed that economic development promotes carbon emissions, while financial development has no significant effect on carbon emissions. To sum up, although the researchers have conducted detailed analysis on the influencing factors of carbon emissions from different perspectives, it is uncommon to analyze the carbon emission reduction via the lens of IA. Especially, IA, as the key factor influencing economic development, has a huge impact on economic growth and environment. Regretfully, the relevant theoretical and empirical research of IA on carbon emissions is still a gap that needs to be filled urgently.

The article "Identifying the Impact of Industrial Agglomeration on China's Carbon Emissions Based on the Spatial Econometric Analysis" was published in 2023. Journal: J Environ Public Health.

The third stream of the literature analyzes the nexus between IA and carbon emissions. With global warming problems gradually becoming more highlighted, IA, as one of the most significant economic development patterns, has received a lot of attention in terms of its impact on environmental pollution, but the results have not yet reached a consensus nowadays. The first view is that IA has a positive environmental externality on carbon emissions. Considering that green technology has been improved through knowledge spillovers and technology spillovers, IA can promote carbon emission reduction. According to Ehrenfeld [32], the establishment of the recycling and sharing of resources among enterprises in the agglomeration regions enhances the efficiency of resource utilization and thus reduces carbon emissions. Using panel data for 14 countries in the G20 during 1991‒2017, Erdoğan et al. [33] studied the impact of agglomeration in industrial sector on carbon emissions, and found that agglomeration significantly inhibits carbon emissions. Zhao et al. [34] employed the 3SLS method to study the influence of producer services' agglomeration on carbon emissions. The findings indicated that producer services' agglomeration has a significant negative effect on carbon emissions in China. In addition, Yan et al. [35] found that financial industry agglomeration can mitigate carbon emission intensity, indicating that an increasing degree of agglomeration may aid in reducing the greenhouse effect. The second view asserts that IA increases regional carbon emissions. This is that excessive agglomeration caused by the congestion effect can accelerate population expansion and energy consumption, and thus promotes total carbon emissions. Virkanen [36] confirmed that IA exacerbates air pollution in southern Finland based on regression analysis. Verhoef and Nijkamp [37] theoretically confirmed that IA causes substantial environmental damage by employing spatial equilibrium model. Chen et al. [38] deliberated agglomeration's influence on the environment and found that an increase in agglomeration exacerbates carbon emissions. Using country-level panel data for 23 OECD countries and 118 non-OECD countries during 1961–2011, Zhang et al. [39] explored the impact of agglomeration on carbon emissions. Their results indicated that industrial agglomeration significantly aggravates carbon emissions. Wu et al. [7] concluded that the scale effect generated by IA would promote carbon emissions in China. Based on panel data of 111 countries in the world during 1982–2017, including Europe Union, North American, East Asia, Nan et al. [40] confirmed that industrial agglomeration has significantly promoted carbon emissions from the perspective of spatial spillover. The third view argues that the linkage between IA and carbon emissions is nonlinear. Specifically, Wang et al. [41] verified that manufacturing agglomeration and carbon emissions have an inverted U-shaped nexus, meaning that carbon emissions will reach the maximum and then steadily decline with the increasing degree of manufacturing agglomeration. The result is also confirmed by Shen and Peng [42]. Moreover, based on Chinese provincial panel data, Liu and Zhang [9] studied the nexus among technological innovation, agglomeration and carbon productivity by using a spatial econometric model. The results exhibited that the nexus between IA and carbon productivity exhibits an inverted U-shaped curve. Using panel data for the top-5 European countries during 1990–2017, Balsalobre-Lorente et al. [43] found that the nexus between energy industry agglomeration and carbon emissions is inverted U-shaped. Meng and Xu [44] used the spatial Durbin model to confirm an inverted N-shaped relationship between industrial collaborative agglomeration and carbon intensity in China. In short, although several scholars discuss the nexus between IA and carbon emissions, few studies have considered the temporal lag effect and the spatial spillover effect. More importantly, most existing literature on the environmental externalities have ignored the effects of different types of IA, which have different theoretical mechanisms and reduction effects on carbon emission.

The article "Identifying the Impact of Industrial Agglomeration on China's Carbon Emissions Based on the Spatial Econometric Analysis" was published in 2023. Journal: J Environ Public Health.

## 3. Theoretical Analysis

This study, which is based on the findings of Copeland and Taylor [45], integrates industrial agglomeration (IA), which is further categorized into specialized agglomeration (SA) and diversified agglomeration (DA), economic growth, and carbon emissions into a unified framework. It then builds a two-sector general equilibrium model that includes households and firms and explores the relationship between IA and carbon emissions.

### 3.1. Production Function

It is assumed that the Cobb–Douglas form, which shows the feature of constant return to scale, can be used to defined the production function of representative firm *i*. The formula is as follows:

(1) $$\begin{array}{c} y_{i}=f\left(K_{i},L_{i}\right)=AK_{i}^{\alpha }L_{i}^{1-\alpha }, \end{array}$$

where *A* is total factor productivity; *K*_i_ and *L*_i_ are the amounts of capital and labor inputs, respectively. The parameter *α* means the capital share of the output, 0 < *α* < 1. When a great number of similar firms congregate in one location, the presence of agglomeration effect prevents the social total production function from simply being the sum of the production functions of all individual firms, and thus, the influence of agglomeration effect on production cannot be ignored. Supposing that the agglomeration function is *G*(·), the expression of social production function is as follows:

(2) $$\begin{array}{c} Y=G\left(•\right)\cdot \overset{n}{\underset{i=1}{\sum }}y_{i}=G\left(•\right)\cdot F\left(K,L\right)=G\left(•\right)\cdot AK^{\alpha }L^{1-\alpha }, \end{array}$$

where *G*(•) reflects the impact of agglomeration on the total social output; *K* and *L* are the total social capital and labor, respectively. Suppose that IA affects the total social output through scale effect, congestion effect, and technological progress, and manifests itself in two types of SA and DA, the agglomeration function is *G*(•) = G(IA) = exp(*ϕ*_1_SA + *ϕ*_2_DA) and the signs of *ϕ*_1_ and *ϕ*_2_ depend on the size of three effects. For simplicity, the social production function is treated in per capita form, then the per capital potential output can be expressed as follows:

(3) $$\begin{array}{c} y=\frac{Y}{L}=G\left(SA,DA\right)\cdot f\left(k\right)=G\left(SA,DA\right)\cdot Ak^{\alpha }\text{,} \end{array}$$

where *y* is the per capital potential output. It is assumed that the society produces a certain amount of carbon emissions while producing product. The increase in carbon emissions will bring negative externalities to the society. When property rights are clearly determined, firms should pay a certain fee for carbon emissions, thus increasing production costs. Therefore, some factors will be used for carbon emission control. Assuming that the proportion of factor inputs used to reduce carbon emissions in the social production process is *θ*, then the per capita real output *x* can be described as follows:

(4) $$\begin{array}{c} x=\left(1-\theta \right)y=\left(1-\theta \right)G\left(SA,DA\right)\cdot f\left(k\right). \end{array}$$

Theoretically, when *θ* equals to 0, it means that the society does not use any inputs to reduce carbon emissions, and the social output will be the potential output *y*; when *θ* is equal to 1, it indicates that the society devotes all essential resources to control carbon emissions, which is inconsistent with reality. In general, the value of *θ* is usually between 0 and 1. Hence, the amount of the social carbon emissions *e* can be presented as follows:

(5) $$\begin{array}{c} e=\phi \left(\theta \right)y=\phi \left(\theta \right)\cdot G\left(SA,DA\right)\cdot f\left(k\right). \end{array}$$

In equation (5), the carbon emission function *φ*(*θ*) = *A*^−1^(1−*θ*)^1/*β*^ is the decreasing function of *θ*, and *φ*′(*θ*) < 0, *φ*″(*θ*) > 0, *β* ∈ [0, 1]. Equation (5) demonstrates that carbon emissions will decrease with the improvement of technology and the increase of investment in carbon emissions control. By combining equations (4) and (5), the real social output function can be further deduced as follows:

(6) $$\begin{array}{c} x=f\left(k,e\right)={\left(Ae\right)}^{\beta }\cdot {\left[G\left(SA,DA\right)\cdot f\left(k\right)\right]}^{1-\beta }\text{,} \end{array}$$

where *e* represents carbon emissions. Equation (6) reveals that the total real output of the society is a compound effect of potential output and carbon emissions.

The article "Identifying the Impact of Industrial Agglomeration on China's Carbon Emissions Based on the Spatial Econometric Analysis" was published in 2023. Journal: J Environ Public Health.

### 3.2. Firms' Production Decision

The purpose of firms' production is profit maximization, which can be realized in two ways. First, given the labor rewards and capital expenditure, firms minimize the production cost of potential output by selecting the optimal capital-labor ratio, which is expressed as follows:

(7) $$\begin{array}{c} C_{y}\left(\omega ,\gamma \right)=\min\;\left\{\left(\omega L+\gamma K\right),G\left(SA,DA\right)\cdot f\left(k\right)=1\right\}, \end{array}$$

where *ω* and *γ* reflect the wage per unit of labor and the return on capital, respectively. By solving the above optimization problem, we can obtain the first-order condition (FOC) as follows:

(8) $$\begin{array}{c} \left.\left(\partial Y/\partial K\right)/\left(\partial Y\right./\partial L\right)=\omega /\gamma \text{.} \end{array}$$

Second, given production cost of potential output and carbon emissions cost, the firms choose the optimal combination of potential output and carbon emissions to minimize the production cost of real output, which can be formulated as follows:

(9) $$\begin{array}{c} C_{x}\left(C_{e},C_{y}\right)=\min\;\left\{\left(C_{e}e+C_{y}y\right),\left(1-\theta \right)\cdot G\left(SA,DA\right)\cdot f\left(k\right)=1\right\}, \end{array}$$

where *C*_y_ is production cost per unit of potential output; *C*_e_ is carbon emission costs; and *C*_x_ is the production cost of real output. By solving the (9), we can obtain the FOC as follows:

(10) $$\begin{array}{c} \left(1-\beta \right)e/\left(\beta y\right)=C_{y}/C_{e}\text{.} \end{array}$$

### 3.3. Corporate Carbon Emissions Decisions

Assuming that the price *p* of the real output *x* is defined exogenously, the total income of firms is *px*. Furthermore, the total cost of firms includes the production cost of potential output *C*_*y*_*y* and the carbon emissions cost *C*_*e*_*e*. Under perfect competition, the long-term profit of firm's production equals to zero, and then, we can obtain as follows:

(11) $$\begin{array}{c} px=C_{y}y+C_{e}e. \end{array}$$

By combining equations (10) and (11), the long-term social carbon emissions can be written as follows:

(12) $$\begin{array}{c} e=\beta px/C_{e}=\beta p\left(1-\theta \right)\cdot G\left(SA,DA\right)\cdot f\left(k\right)/C_{e}\text{.} \end{array}$$

### 3.4. Social Welfare Maximization

As shown by Grimaud and Rouge [46], the social welfare function *U*(*x*, *e*) is as follows:

(13) $$\begin{array}{c} U\left(x,e\right)=x^{1-\varepsilon }/\left(1-\varepsilon \right)-e^{1+\rho }/\left(1+\rho \right)\text{,} \end{array}$$

where *ε* is the coefficient of relative risk aversion, *ρ* is the degree of social desire for carbon emissions, and *ε* > 0, *ρ* > 0. Assume that there is a social rule maker who decides on output *x* and carbon emissions *e* to maximize social welfare, the FOC of utility maximization can be derived as follows:

(14) $$\begin{array}{c} \left(\partial U/\partial x\right)\cdot \left(\partial x/\partial e\right)=e^{\rho }. \end{array}$$

Notably, the marginal cost of carbon emissions matches the marginal benefit of real output under the assumption that property rights are clearly defined, or ∂*U*/∂*x* = ∂*x*/∂*e*, and then it can be flattened by inserting it into equation (14) to yield the following:

(15) $$\begin{array}{c} C_{e}=\frac{\partial x}{\partial e}=e^{\rho /2}\text{.} \end{array}$$

Finally, by combing formulas (12) and (15), the social carbon emissions in long-term equilibrium can be further sorted out as follows:

(16) $$\begin{array}{c} e={\left[A\beta \rho \left(1-\theta \right)\right]}^{2/\left(\rho +2\right)}\cdot G{\left(SA,DA\right)}^{2/\left(\rho +2\right)}\cdot k^{2\alpha /\left(\rho +2\right)}. \end{array}$$

Let *μ* = *Aβp*(1 − *θ*), *π* = 2/(*ρ* + 2), then equation (16) can be further simplified as follows:

(17) $$\begin{array}{c} e=\mu^{\pi }\cdot G\left(S\right.A,DA{}^{\left(\pi \right)}\cdot k^{\alpha \pi }=\mu^{\pi }\cdot \exp\;\left(\varphi_{1}\right.\pi SA+\varphi_{2}\pi D\left.A\right)\cdot k^{\alpha \pi }. \end{array}$$

After taking the logarithm of both sides of equation (17), the following expression can be obtained:

(18) $$\begin{array}{c} \ln\;e=\pi \cdot \ln\;\mu +\varphi_{1}\pi \cdot SA+\varphi_{2}\pi \cdot DA+\alpha \pi \cdot \ln\;k. \end{array}$$

Equation (18) reveals that IA primarily influences carbon emissions through knowledge spillover or resource restrictions brought on by the externalities of SA and DA. Hence, the purpose of this study is to explore the impact of two different types of agglomeration on carbon emissions.

The article "Identifying the Impact of Industrial Agglomeration on China's Carbon Emissions Based on the Spatial Econometric Analysis" was published in 2023. Journal: J Environ Public Health.

## 4. Methodology, Variables Selection, and Data Sources

Based on the theoretical analysis, it is obvious that IA affects carbon emissions through different pathways, and the sign of the impact has greater uncertainty. To deeply investigate the nexus between IA and carbon emissions, some empirical models used for the analysis are built in this study.

### 4.1. Specification of the Dynamic Nonspatial Econometric Model

First, we construct a dynamic nonspatial panel model to analyze the nexus between IA and carbon emissions. Since present carbon emissions may be affected by previous carbon emission, the first-order lag term of carbon emissions is also incorporated into the model as an explanatory variable to reflect the dynamic cumulative effect of carbon emissions. The model is depicted as follows:

(19) $$\begin{array}{c} \ln\;CE_{it}=\gamma \;\ln\;CE_{it-1}+\delta \;\ln\;IA_{it}+\beta X_{it}+\mu_{i}+\lambda_{t}+\varepsilon_{it}\text{,} \end{array}$$

where the subscripts *i* and *t* is the province and year, respectively, and *CE*_*it*_ represents per capita carbon emissions. *CE*_*it*−1_ stands for the first-order lag term of *CE*_*it*_ as an explanatory variable. IA denotes industrial agglomeration, which is classified into SA and DA in empirical analysis. *X* represents a set of control variables, including economic development (pgdp), environmental regulation (er), urbanization rate (ur) and infrastructure (inf), respectively. Meanwhile, *γ* denotes the time-lagged coefficient of carbon emissions. *β* represents the coefficients of the control variables to be estimated. In addition, *μ*_*i*_, *λ*_*t*_, and *ε*_*it*_ denote individual effect, time effect, and random error term, respectively.

### 4.2. Specification of the Spatial Dynamic Panel Model

According to the First Law of Geography, economic matters in a certain area have significant spatial dependence, and the closer the geographical distance is, the stronger the spatial connection is [47, 48]. Obviously, carbon emissions are not just a local environmental issue, they may also spread to the adjacent regions due to factors including atmospheric circulation and industrial transfer, and thus, the spatial spillover effects need to be considered when we explore the elements that influence interprovincial regional carbon emissions in China. With this in mind, following Elhorst [49], this study uses the dynamic spatial lag panel model to investigate the effects of SA and DA on carbon emissions. The dynamic spatial panel lag model developed in this study can be described as follows:

(20) $$\begin{array}{c} \ln\;CE_{it}=\gamma \;\ln\;CE_{it-1}+\rho W\;\ln\;CE_{it}+\eta W\;\ln\;CE_{it-1}+\delta \;\ln\;IA_{it}+\beta X_{it}+\mu_{i}+\lambda_{t}+\varepsilon_{it}\text{,} \end{array}$$

where *W* represents a spatial weight matrix. The variables WlnCE_it_ and WlnCE_it−1_ denote the carbon emissions of the neighboring regions in the current and previous periods, respectively. *γ*, *ρ*, *η*, *δ*, and *β* stand for the regression coefficients to be estimated. Among them, *γ* denotes the time lag coefficient, capturing the effect of previous carbon emissions on current carbon emissions; *ρ* is the spatial lag coefficient, reflecting the effect of other provinces' carbon emissions on the sample provinces in the current period, *η* is the spatiotemporal lag coefficient, indicating the influence of other provinces' previous carbon emissions on the sample provinces. Most notably, in the model (20), when *δ* is significantly more (less) than 0, which means that IA aggravates (curbs) carbon emissions. To assure the consistency and validity of the empirical findings, this study employs the maximum likelihood method to estimate the abovementioned model.

The article "Identifying the Impact of Industrial Agglomeration on China's Carbon Emissions Based on the Spatial Econometric Analysis" was published in 2023. Journal: J Environ Public Health.

Furthermore, the essential issue of the spatial econometric model is how to depict the spatial linkage across areas, that is, how to construct a spatial weight matrix. Geographical adjacency, geographical distance, economic distance and economic distance for the specification of spatial weight matrix are the four most common forms in the existing literature. Taking the availability and integrity of data into consideration, we use the geographical adjacency weight matrix (W1), economic geographic distance weight matrix (W2), and economic geography nested weight matrix (W3) to estimate the model (20). To be specific, the adjacency weight matrix is determined by whether the provinces are geographically contiguous or not. The weight is set to 1 if two provinces are contiguous; otherwise, it is put to 0, and the diagonal components are set to 0. However, the economic geographical distance weight matrix and economic geography nested weight matrix are constructed according to the geographic distance and economic development level. The method to construct a matrix can be divided into three steps. First, this paper calculates the geographical distance among provinces using the longitude and latitude, and measures the reciprocal of the geographical distance to obtain the geographical distance weight matrix. Second, based on the level of economic development of each province, the economic weight matrix is created. Third, by using the above two matrices and a certain algorithm, we establish the economic geographic distance matrix and economic geographic nested matrix, respectively. Most notably, if the original data of the weight matrix are obtained, each weight matrix is further standardized, indicating that the sum of each row in each matrix is equal to 1.

### 4.3. Variable Selection and Data Sources

#### 4.3.1. Dependent Variable

The explained variable is carbon emissions per capita (CE). Although most developed countries have released relevant data on carbon emissions, the official data are still unpublished in China, and its measurement has always been a difficult problem in academic circles. The current mainstream views believe that carbon emissions are mostly from the burning of fossil fuels and the production of cement [50]. Therefore, we also use this method to measure the scale of carbon emissions for each province. Specifically, carbon dioxide produced by fossil fuel combustion mainly comes from the following seven types: gasoline, coal, coke, diesel, kerosene, fuel oil, and natural gas, while carbon dioxide produced by cement production comes from the industrial sector. The formula for calculating carbon emissions is as follows:

(21) $$\begin{array}{c} CE_{it}=\sum_{k=1}^{7}E_{itk}\times S_{k}\times C_{k}+Q_{it}\times C_{\text{cement}}\text{,} \end{array}$$

where the subscripts *i* and *t* are province and year, respectively, and *k* stands for the type of energy. CE_*it*_ denotes the carbon emission for the *t* year in *i* province. *E*_*itk*_, *S*_*k*_, and *C*_*k*_ represent the standard coal conversion coefficient, carbon emission coefficient, and the amount of the *k*-th fossil energy consumed, respectively. *Q*_*it*_ and *C*_cement_ reflect the carbon emission factor and the quantity of cement production. In equation (21), the requirements for the carbon emission coefficient and the standard coal conversion coefficient are taken from the National Greenhouse Gas Emission Inventory (2006) published by the IPCC. *E*_*itk*_ × *S*_*k*_ × *C*_*k*_ measures the amount of carbon emissions from fossil fuels burning, and *Q*_*it*_ × *C*_cement_ denotes the amount of carbon emissions from cement production. Moreover, to eliminate the impact of population scale on the estimation results, we use the ratio of total carbon emissions to the population of each province as the explained variable.

The article "Identifying the Impact of Industrial Agglomeration on China's Carbon Emissions Based on the Spatial Econometric Analysis" was published in 2023. Journal: J Environ Public Health.

#### 4.3.2. Core Independent Variables

In order to achieve economies of scale and reduce production costs, firms that be characterized by similar product structures or relevant industrial chains are prone to gather in the same geographic area, thus IA is mainly manifested in two forms: SA and DA [51].

Specialized agglomeration (SA). SA refers to the concentration of industries with homogeneous input and output in a specific geographic region, which distorts the allocation of production factors and causes a single industrial structure, and then, stimulates the carbon emissions. The formula for SA is as follows:

(22) $$\begin{array}{c} SA_{i}=\max\;\left(w_{ij}/w_{j}\right). \end{array}$$

Diversified agglomeration (DA). DA includes horizontal agglomeration with technology linkage and vertical agglomeration with the upstream and downstream relationship of the industrial chain. Generally, DA promotes the sharing of knowledge, technology, and basic equipment, which further improves the level of green technology development and the efficiency of energy, and curbs carbon emissions ultimately. The formula for DA is as follows:

(23) $$\begin{array}{c} DA_{i}=1/\sum \left(w_{ij}/w_{j}\right)\text{.} \end{array}$$

In equations (22) and (23), *i* and *j* is the regions and industry, respectively, *w*_*ij*_ is the employment rate of industry *j* in region *i*, and *w*_*j*_ is the national employment rate of industry *j*. The greater the value of the index, the deeper the degree of regional IA.

The article "Identifying the Impact of Industrial Agglomeration on China's Carbon Emissions Based on the Spatial Econometric Analysis" was published in 2023. Journal: J Environ Public Health.

#### 4.3.3. Control Variables

In order to mitigate the endogenous problem caused by omitted important variables and to increase the accuracy of the regression results, five control variables are included in the model by referring to previous literature. Details of the control variables are shown below.

Per-capita GDP (pgdp). Some researchers confirmed that the degree of economic progress and carbon emissions are highly correlated [30]. Specifically, a region with higher economic development tends to have greater demand for energy consumption, which in turn increases carbon emissions. In this paper, the indicator is calculated by the ratio of gross domestic product to population, which is considered one of the control variables.

Environmental regulation (er). The government can regulate the production mode of enterprises by using reasonable environmental supervision, so as to effectively stimulate the innovation enthusiasm of enterprises in green energy-saving technology and decrease the need for fossil energy and promote carbon emission reduction [25]. In order to explore the influence of environmental regulation on carbon emissions, we choose the ratio of total investment in industrial pollution control to the total population as a proxy variable for analysis. In addition, the squared term of environmental regulation is also incorporated into the regression model to study the probable nonlinear link between the two [52].

Urbanization rate (ur). Theoretically, compared with rural areas, there are more modern infrastructure and fossil fuel consumption in urban areas, thus emitting more carbon dioxide. Actually, the higher the degree of agglomeration in urban areas is, the greater the benefits of increasing returns to scale in energy use, such as convenient transportation and centralized heating supply, which is beneficial to reduce carbon emissions [53]. Therefore, the ratio of the urban population is used to represent urbanization for each region.

Infrastructure (inf). Infrastructure should be included in the model to reflect its impact on regional carbon emissions and environmental quality by reducing energy use and transaction costs while boosting efficiency per unit of energy used [50, 54]. In this paper, the ratio of road miles to population is used to represent infrastructure.

The article "Identifying the Impact of Industrial Agglomeration on China's Carbon Emissions Based on the Spatial Econometric Analysis" was published in 2023. Journal: J Environ Public Health.

### 4.4. Data Source

Considering the availability of sample data and the actual needs of research, this study utilizes a balanced panel data set of 30 provinces in mainland China (excluding Tibet, Macao, Hong Kong, and Taiwan) to empirically investigate the effects of different industrial agglomeration patterns on carbon emissions. Specifically, the China Energy Statistical Yearbook included the data on fossil fuels and cement production. The China Industrial Economic Statistical Yearbook provided the data for the IA. The data on the environmental regulation are collected from China Environment Statistical Yearbook. Other variables are collected and compiled from the Provincial Statistical Yearbook of each province. In addition, the moving average and interpolation methods are used to supplement the missing data in the study. Furthermore, all absolute value variables, except for the urbanization rate, are changed into logarithmic forms to remove heteroscedasticity. Meanwhile, in order to eliminate the price effect, we use a CPI index to deflate all nominal variables to real variables based on the 2003 constant price. The descriptive statistics for all variables are shown in Table 1.

## 5. Empirical Results and Analysis

### 5.1. Panel Unit Root Test

Before conducting the empirical analysis, the panel stationarity test is performed on all variables to eliminate spurious regression problems. To be specific, this paper adopts four stationarity test methods, namely, Levin–Lin–Chu (LLC), Im–Pesaran–Shin (IPS), Augmented Dickey–Fuller Fisher (ADF-Fisher), and Phillip Perron Fisher (PP-Fisher) tests to determine stationarity, and the results are shown in Table 2. The results reveal that each variable's raw data sequence is stationary. Furthermore, this paper employs the variance inflation factor (VIF) test for the sake of eliminating the multi-collinearity problem, and the findings are presented in Table 2, Column 6. VIF has a minimum and maximum values of 1.13 and 6.34, respectively, which are less than the critical threshold of 10, suggesting that multi-collinearity among the variables is not a severe issue.

### 5.2. Preliminary Regression Results

The objective of this paper is to investigate the effects of SA and DA on carbon emissions. First, we adopt the traditional nonspatial model to explore the relationship between agglomeration and carbon emissions, which is a preliminary empirical analysis. Specifically, this paper uses five methods to estimate (19), including FGLS, RE, FE, DIFF-GMM, and SYS-GMM. The results are shown in Table 3. It is worth noting that the statistical values of the serial autocorrelation test (as shown by the *p* values of AR test) and the overidentification test (see the *p* values of the Hansen test) show that the selection of model instrumental variables is reasonable, and the results of generalized method of moments estimation are reliable. In addition, the coefficients of SA and DA are also similar in sign and significance among the five estimation models, suggesting that the results of the empirical evidence are robust.

The article "Identifying the Impact of Industrial Agglomeration on China's Carbon Emissions Based on the Spatial Econometric Analysis" was published in 2023. Journal: J Environ Public Health.

In Table 3, the impact of SA on carbon emissions shows a significant positive relationship, while the impact of DA on carbon emissions has a significant negative link. That is to say, an increasing degree of SA promotes carbon emissions, while an improvement in DA level could help China reduce carbon emissions. In addition, the level of economic development has a significantly positive link with carbon emissions, and environmental regulation and carbon emissions have a significant inverted U-shaped relationship, whereas urbanization and infrastructure have a positive influence on carbon emissions. Furthermore, the coefficient of lagged carbon emissions is also significantly positive, indicating that carbon emissions have a significant positive inertia over time.

### 5.3. Analysis from the Spatiotemporal Perspective

Since there may be considerable spatial correlations in China's regional carbon emissions, the spatial dynamic econometric model is used to account for both the spatial and dynamic effects in order to assure more effective results.

#### 5.3.1. Spatial Autocorrelation Test

We must first determine whether there is a spatial correlation between provincial carbon emissions in China before proceeding with a spatial econometric analysis. Given the vast size of China, there are significant regional differences in the level of economic development; this paper draws quartile maps of carbon emissions in the years of 2003 and 2019, as shown in Figure 2, to visually reflect the spatial distribution features and spatiotemporal evolutionary features in carbon emissions. China's provincial carbon emissions, according to the maps, reveal both regional heterogeneity and spatial clustering. On the one hand, the degree of carbon emission in the eastern, central, and western regions are obvious differences. Regional carbon emissions, on the other hand, exhibit clear positive agglomeration, i.e., carbon emissions exhibit high-high agglomeration and low-low agglomeration. In addition, the level of carbon emissions in China gradually increases from 2003 to 2019. In order to obtain the statistical significance of the spatial autocorrelation of carbon emissions, we further employ empirical methods to conduct a related study.

There are three main methods for testing spatial correlation in practice, namely, Getis–Ord's *G* test, Geary's C test, and Moran's I test. Among them, Moran's I test is the most widely used approach in academic circles. In view of this, following Moran [55], this paper employs the global Moran's I test to demonstrate the spatial autocorrelation and agglomeration of China's province-level carbon emissions. The following formula can be used to determine the global Moran's I index:

(24) $$\begin{array}{c} {Moran}^{\prime }sI=\frac{n\sum_{i=1}^{n}\sum_{j=1}^{n}W_{ij}\left(CE_{i}-\bar{CE}\right)\left(CE_{j}-\bar{CE}\right)}{\sum_{i=1}^{n}\sum_{j=1}^{n}W_{ij}\sum_{i=1}^{n}{\left(CE_{i}-\right)}^{2}}, \end{array}$$

where CE_*i*_ and CE_*j*_ are the per capita carbon emissions of provinces *i* and *j*, respectively, and represent the average values of CE; *W*_*ij*_ represents the constituent elements of the spatial weight matrix, located in the *i*-th row and *j*-th column, and *n* stands for the number of provinces.  Table 4 displays the results of the global Moran's I test for China's carbon emissions from 2003 to 2019 by using three weight matrices. The results display that the values of Moran's I of carbon emissions are significantly positive, which means that provinces with a similar degree of carbon emissions are clustered together, i.e., high emitting provinces are adjacent to each other or low emitting provinces are adjacent to each other. Therefore, considering the importance of spatial autocorrelation, the spatial econometric model is adopted to eliminate the estimated bias caused by traditional panel models.

The article "Identifying the Impact of Industrial Agglomeration on China's Carbon Emissions Based on the Spatial Econometric Analysis" was published in 2023. Journal: J Environ Public Health.

#### 5.3.2. Baseline Regression Result

The main objective of our paper is to explore the effect of SA and DA on carbon emissions by using the dynamic spatial lag model. Specifically, the Hausman test is used to choose the fundamental form of the spatial panel model, and the findings indicate that the two-way fixed effect model (FE) should be considered. Then, we introduce the three spatial weight matrices above and employ the maximum likelihood method to estimate the (20). The baseline regression results of the geographic adjacency weight matrix (W1), economic geographic weight matrix (W2), and economic geographic nesting weight matrix (W3) are shown in Table 5. The results take into account the dual effects of economic development level and geographical distance on regional spatial association.

First, the study explores the temporal and spatial evolution characteristics of carbon emissions, and the results show that carbon emissions featured a double lag impact in both time and space. To be specific, the coefficients of lnCE_it−1_ (*γ*) are positive in all models and significant at the 1% level, suggesting that carbon emissions have a significant positive lagged effect in the time dimension. If carbon emissions are quite high in the present time, carbon emissions in the following period will continue to climb, and a cumulative impact of carbon emissions may emerge. Furthermore, the coefficients of *W* × lnCE_it_ (*ρ*) are all significant and positive, fully manifesting that carbon emissions have a remarkable spatial agglomeration effect. The main manifestation is that an increase in emissions concentration of neighboring provinces will aggravate the levels of carbon emissions of the sample province. This might be attributed to natural atmospheric movement, industry linkage, economic intercourse, and regional replication of environmental laws. Moreover, the coefficients of *W* × lnCE_it−1_ (*η*) are significantly negative in all models, indicating that the high carbon emissions degree of the surrounding provinces in the previous period can significantly decrease the current emissions level of the sample province. One feasible explanation is that as the central government has gradually strengthened efforts to supervise the environment among regions when formulating carbon emission policies in their jurisdictions, local governments must not only take into account the local level of green economic development but also assess the degree of carbon emission in neighboring regions, to gain more political promotion benefits in environmental governance.

The article "Identifying the Impact of Industrial Agglomeration on China's Carbon Emissions Based on the Spatial Econometric Analysis" was published in 2023. Journal: J Environ Public Health.

Second, we further investigate the effects of SA and DA on carbon emissions. In terms of SA, its coefficients are significantly positive in all models, which demonstrates that the improved level of SA has significantly promoted carbon emission. We can summarize the reasonable explanations into the following two aspects. As the industries with homogeneous inputs and outputs continue to cluster in a region, the “congestion effect” occurs when production factors are overly concentrated, disrupting the factor market's order. On the one hand, factor distortion reduces overall factors utilization efficiency and increases fossil energy consumption to aggravate the pollution discharge load, which exceeds the regional environmental carrying capacity and causes an increase in carbon emissions ultimately. On the other hand, ruthless competition among firms hinders the spillover of energy-saving and emission-reduction technology and knowledge, which weakens the motivation for innovation in technology and prevents technological progress, which results in high carbon emissions and resource waste per unit of output. In terms of DA, its coefficients are all significant and negative, indicating that the increase in the level of DA has significantly curbed carbon emissions. Actually, DA has an impact on carbon emissions through the scale effect and the effect of technology spillover. Notably, DA brings more heterogeneous knowledge, which is favorable to promote innovation in technology and improve production efficiency and thus effectively reduce carbon emissions. In addition, DA realizes the recycling and sharing of resources and infrastructure among firms, which is helpful to achieve scale economies and improve resource utilization efficiency, and curbs carbon emissions in agglomeration areas eventually.

The article "Identifying the Impact of Industrial Agglomeration on China's Carbon Emissions Based on the Spatial Econometric Analysis" was published in 2023. Journal: J Environ Public Health.

Third, we analyze the impacts of control variables on carbon emission. Specifically, the regression coefficients of per capita GDP are generally positive but not significant in all models, indicating that China's economic development is weakly decoupled from carbon emissions. The possible explanation is that although the governments actively promote green and low-carbon development, due to the limitations of technological innovation capability and industrial structure adjustment, environmental pollution control efforts are relatively small, so the decoupling effect of economic development and carbon emissions is not obvious. The conclusion is also supported by Gao et al. [56] and Liu et al. [57]. In addition, the impact of environmental regulation on carbon emissions exhibits a nonlinear relationship, namely, an inverted U-shaped nexus. As the degree of environmental regulation is gradually strengthened, its effect on carbon emissions changes from an aggravating effect to an emission reduction effect. Moreover, the coefficient of urbanization is significantly negative on the whole, demonstrating that an increase in urbanization can curb carbon emissions. Due to the rapid development of urbanization in the past decades, the new-type urbanization may bring greater scale effects and less energy needs, resulting in carbon emissions reduction. Additionally, there is a significant negative impact of infrastructure on carbon emissions, which means that the improvement of infrastructure level can meet the desired carbon reduction target. A plausible explanation is that infrastructure can reduce carbon emissions by reducing transport and transaction costs and increasing total factor productivity.

### 5.4. Regional Heterogeneity Analysis

According to the regression results for the full sample, the effect of SA on carbon emissions is significantly positive, whereas the impact of DA is negative. However, due to the step-by-step development strategy of China's regional economy, there are large differences in carbon emission levels and industrial development in various regions of China. Is there a regional heterogeneity in the effect of SA and DA on carbon emissions? To gain insights into regional heterogeneity, the full sample is divided into three subsamples, namely, eastern, central, and western regions, based on the geographic location and level of economic development. Then, this study uses the dynamic spatial econometric method to explore the impacts of SA and DA on carbon emissions for three subsamples, respectively. The heterogeneity regression results are shown in Table 6.

The article "Identifying the Impact of Industrial Agglomeration on China's Carbon Emissions Based on the Spatial Econometric Analysis" was published in 2023. Journal: J Environ Public Health.

First, we analyze the regional heterogeneity in the impact of SA on carbon emissions. Specifically, the sign of the coefficient of SA is positive but insignificant in the eastern region. The conceivable explanation is that the local governments develop the concept of green development while focusing on industrial development. Moreover, the economic growth is progressively changing from an extensive mode to an intensive mode in the eastern region, which weakens the effect of SA in promoting carbon emissions. In addition, the SA coefficient is significantly positive in the central and western areas, and the sign and significance are in line with the baseline test results. Second, this study probes the regional heterogeneity in the influence of DA on carbon emissions. Specifically, the coefficient of DA is negative and insignificant in the eastern and central areas. The reasons can be summarized as follows: the long-term priority of industrial development in the eastern provinces leads to a low proportion of the primary and secondary industries and a low degree of inter-industry coupling, which ultimately nullifies the emission reduction effect of DA. Furthermore, the coefficient of DA is notably negative in the western region, implying that DA can effectively curb carbon emissions, which is in line with the baseline regression results. In summary, the significance of coefficients is slightly different among regions, which verifies the existence of regional heterogeneity.

### 5.5. Robustness Test

To assure the robustness, reliability, and consistency of the baseline regression results, the study implements robustness tests from three aspects. First, we adjust the sample period by intercepting the sample data for two years to remove the effect of sample outliers. Next, we replace the measurement methods of carbon emissions. To be specific, we use the ratio of the total carbon emissions to gross domestic product as a substitution variable for robustness analysis and then analyze the adjusted data. Finally, except for the three spatial weight matrices mentioned above, the economic distance weight matrix is used to further verify the robustness of the conclusion [58]. The regression results of the three robustness methods are shown in Table 7.

The article "Identifying the Impact of Industrial Agglomeration on China's Carbon Emissions Based on the Spatial Econometric Analysis" was published in 2023. Journal: J Environ Public Health.

Columns (1) and (2) in Table 7 report the regression results for adjusting the sample period, demonstrating that SA promotes carbon emissions, while DA significantly inhibits the carbon emissions. In addition, carbon emissions have significant lag effects and spatial spillover effects. Columns (3) and (4) in Table 7 show the results of remeasuring the carbon emissions, suggesting that SA has a significantly positive impact on carbon emissions, while the influence of DA is significantly negative. After remeasuring the index of carbon emissions, the coefficients of each variable have the same signs and significance as the benchmark regression findings. Columns (5) to (6) in Table 7 show the results of replacing the weight matrix, showing that the degree of SA is positively correlated with the level of carbon emissions, while the degree of DA is negatively correlated. Moreover, the differences in other variables are not obvious, revealing that the main conclusions of replacing the weight matrix are in line with the benchmark empirical analysis. In summary, the robustness analysis verifies that the carbon emissions have path-dependent effects and spatial spillover effects, and the consequences of various forms of IA on carbon emissions are vastly varied. Moreover, the signs of all control variables are in line with the baseline regression results. The robustness test results are highly similar to the baseline regression results, which confirm the baseline regression results are robust and reliable.

## 6. Conclusions and Policy Recommendations

Excessive carbon emissions make economic development unsustainable, and the precise identification of driving factors of carbon emissions is an important precondition to implementing targeted emissions reduction policies. Under such circumstances, this study constructs a two-sector general equilibrium model to analyze the theoretical mechanism of IA on carbon emissions. Then, we find that IA mainly affects carbon emissions through agglomeration effects and congestion effects. Based on the theoretical analysis, this study explores the relationship between two different types of IA and carbon emissions by employing the dynamic spatial lag model and the sample data of 30 Chinese provinces from 2003 to 2019. The findings of the spatial econometric model can be concluded as follows. First, under different spatial weight matrices, carbon emissions have significant path dependence characteristics in the time dimension, positive correlation, and agglomeration in the space dimension and restrain the carbon emissions of adjacent regions in the next period in the space and time dimension. Second, there is a strong link between IA and carbon emissions. Among them, SA has a significant positive impact on carbon emissions, while DA has a negative impact. Third, environmental regulation and carbon emissions have an inverted U-shaped link, whereas urbanization and infrastructure have a negative link with carbon emissions, and economic development is weakly decoupling from carbon emissions. Finally, at the regional level, the significance of the coefficients of SA and DA differ among the three regions, indicating the existence of regional heterogeneity.

The article "Identifying the Impact of Industrial Agglomeration on China's Carbon Emissions Based on the Spatial Econometric Analysis" was published in 2023. Journal: J Environ Public Health.

In order to achieve high-quality development, we provide some feasible suggestions for reducing carbon emissions and promoting the healthy development of IA based on the abovementioned results.

First, China should promote the green and low-carbon development approach, as well as energy conservation and emission reduction. Specifically, the government should enhance its support for green energy and encourage the upgrading of the energy consumption structure. Accelerating the promotion and use of clean energy is conducive to reducing the use of nonrenewable and heavily polluting energy, as well as reducing carbon emissions from the source. Simultaneously, environmental assessment should be implemented into the performance evaluation system of local governments to provide a long-term mechanism for emission reduction. In addition, only by crossing the barriers of administrative divisions and establishing a resource-sharing platform and cooperative projects for governance among regions could the long-term mechanism of carbon emissions reduction be achieved. Strengthening interprovincial collaboration and promoting joint governance is critical. Finally, the “one-size-fits-all” policy paradigm is unsuitable for China's current situation which requires consideration of the special attributes of economic level and resource endowments. Differentiated development strategies for carbon emissions reduction should be tailored to the needs of China's various regions.

Second, the Chinese government should prolong the industry chain and promote industrial DA. Specifically, through policy support and tax incentives, the government guides local enterprises to form DA areas and realize the rationalization of the industrial structure. The government should promote enterprises to strengthen cooperation, speed up the movement of labor, information, knowledge, and technology among regions, and make full use of the emission reduction effect of the positive externality of DA. In addition, the government should encourage SA to carry out diversified structural adjustments, cultivate connected supporting industries on the basis of existing industries, prolong the industry chain, and promote enterprises to curb carbon emissions. Finally, when the congestion effect of IA begins to appear, the industrial transfer should be carried out to reduce the adverse influence of excessive clustering on the environment and achieve the sustainable development of the economy and environment.

The article "Identifying the Impact of Industrial Agglomeration on China's Carbon Emissions Based on the Spatial Econometric Analysis" was published in 2023. Journal: J Environ Public Health.

Third, to achieve China's “dual carbon” goal, we should take advantage of the synergistic impacts of economic development, environmental supervision, urbanization, and infrastructure to reduce carbon emissions. Specifically, (1) while developing the economy, we should pay attention to carbon emission reduction and environmental protection., accelerate the transition from an extensive to an intensive economy mode, achieve a balance between regional economic growth and carbon emissions, and achieve sustainable economic development. (2) The administration ought to tighten environmental regulations, add investments in emissions pollution control, mobilize social funds, and provide financial support for carbon emission reduction. (3) We should accelerate the construction of new urbanization with energy-saving and emission reduction as the core, speed up the layout of city that is compatible with the carrying capacity of resources and the environment, and take a new urbanization path that is intensive, intelligent, low in carbon, and green. (4) The state and local governments should improve infrastructure construction, which aids in the improvement of energy efficiency and the reduction of carbon emissions.

### 6.1. Limitations and Outlook

The effect of different types of IA on the performance of regional carbon emissions in China is the focus of this paper. Although this study gives useful information, it does have several shortcomings that might be addressed in future studies. First, although this paper empirically analyzes the different effects of SA and DA on carbon emissions based on a dynamic spatial perspective, their impact mechanism and dynamic evolutionary process have not been adequately explored due to the limitation of sample data. Therefore, the subsequent research will try to develop a dynamic stochastic general equilibrium (DSGE) model to describe the transmission mechanisms of IA on carbon emissions and provide empirical evidences to deepen this study [59]. Second, as the measurement of carbon emissions has always been the focus of academic debate, carbon emissions from seven kinds of fossil fuel combustion and cement production are used to measure the dependent variable in the study. Due to the unavailability of relevant data, this paper only calculates the scale of carbon emissions at the provincial level and does not involve the prefecture (or industry) level [60]. Specifically, as different prefectures (or industries) in the same province have different levels of economic development, once the sample data at the prefecture (or industry) level can be obtained in the future, we can explore the effect of IA on carbon emissions at prefecture (industry) level and significantly improve the empirical research due to the expansion of the sample size.

The article "Identifying the Impact of Industrial Agglomeration on China's Carbon Emissions Based on the Spatial Econometric Analysis" was published in 2023. Journal: J Environ Public Health.

## Figures and Tables

**Figure 1:** Trends of energy consumption, carbon emissions, and GDP growth rate in China. Figure 1 is reproduced from Xu and Li [3], (under the creative commons attribution license/public domain).

**Figure 2:** Spatial distribution of Chinese provincial carbon emissions in 2003 and 2019 (unit: tons per capita).

**Table 1:** Descriptive statistics for all variables from 2003 to 2019.

Definition	Symbol	Mean	Std. dev	Min	Max	Obs
Carbon emissions	lnCE	1.672	0.559	0.266	3.988	510
Specialized agglomeration	lnSA	0.304	0.190	0.018	0.780	510
Diversified agglomeration	lnDA	1.591	0.778	0.219	4.494	510
Per-capita gross domestic product	lnpgdp	10.046	0.642	8.218	11.663	510
Environmental regulation	lner	3.291	0.815	0.769	5.612	510
Urbanization rate	ur	0.527	0.143	0.248	0.896	510
Infrastructure	lninf	0.982	0.651	−1.000	2.653	510

**Table 2:** Results of unit root tests and VIF test.

Variable	LLC	IPS	ADF-Fisher	PP-Fisher	VIF
lnCE	−3.252^*∗∗∗*^	−1.359^*∗*^	115.609^*∗∗∗*^	442.049^*∗∗∗*^	‒
lnSA	−2.071^*∗∗*^	−2.265^*∗∗*^	89.938^*∗∗∗*^	89.611^*∗∗∗*^	1.15
lnDA	−3.849^*∗∗∗*^	−1.996^*∗∗*^	105.835^*∗∗∗*^	120.416^*∗∗∗*^	1.14
lnpgdp	−4.711^*∗∗∗*^	−1.441^*∗*^	78.727^*∗∗*^	471.883^*∗∗∗*^	5.75
lner	−7.095^*∗∗∗*^	−4.781^*∗∗∗*^	84.926^*∗∗*^	145.578^*∗∗∗*^	1.13
ur	−5.021^*∗∗∗*^	−1.695^*∗∗*^	165.565^*∗∗*^	173.195^*∗∗∗*^	6.34
lninf	−4.623^*∗∗∗*^	−7.749^*∗∗∗*^	95.827^*∗∗∗*^	170.943^*∗∗∗*^	1.44

^*∗∗∗*^, ^*∗∗*^, and ^*∗*^ represent significance at 1%, 5%, and 10% levels, respectively.

**Table 3:** Non-spatial panel regression results of impact of SA and DA on carbon emissions.

Variable	*FGLS*		*RE*		*FE*		*DIFF-GMM*		*SYS-GMM*	
	(1)	(2)	(3)	(4)	(5)	(6)	(7)	(8)	(9)	(10)
L.lnCE							0.265^*∗∗*^	0.236^*∗*^	0.284^*∗∗∗*^	0.209^*∗*^
							(0.123)	(0.135)	(0.087)	(0.127)
lnSA	0.126^*∗*^		0.601^*∗∗∗*^		0.815^*∗∗∗*^		0.604^*∗∗*^		0.232^*∗∗*^	
	(0.073)		(0.085)		(0.085)		(0.299)		(0.114)	
lnDA		−0.038^*∗∗*^		−0.078^*∗∗∗*^		−0.097^*∗∗∗*^		−0.106^*∗∗*^		−0.144^*∗*^
		(0.018)		(0.021)		(0.021)		(0.050)		(0.082)
lnpgdp	0.064	0.071	0.193^*∗∗∗*^	0.215^*∗∗∗*^	0.102	0.243^*∗∗∗*^	0.577^*∗∗∗*^	0.572^*∗∗∗*^	−0.295^*∗∗∗*^	0.388^*∗*^
	(0.057)	(0.056)	(0.055)	(0.057)	(0.082)	(0.087)	(0.145)	(0.138)	(0.079)	(0.219)
lner	0.087	0.090	0.216^*∗∗∗*^	0.197^*∗∗∗*^	0.193^*∗∗∗*^	0.183^*∗∗∗*^	0.638^*∗∗∗*^	0.485^*∗∗∗*^	0.022	0.555^*∗∗∗*^
	(0.058)	(0.058)	(0.059)	(0.061)	(0.053)	(0.057)	(0.188)	(0.184)	(0.069)	(0.140)
[lner]^2^	−0.002	−0.002	−0.020^*∗∗*^	−0.016^*∗*^	−0.018^*∗∗*^	−0.016^*∗*^	−0.089^*∗∗∗*^	−0.068^*∗∗*^	0.006	−0.078^*∗∗∗*^
	(0.009)	(0.009)	(0.009)	(0.010)	(0.008)	(0.009)	(0.027)	(0.026)	(0.011)	(0.022)
ur	1.592^*∗∗∗*^	1.568^*∗∗∗*^	0.753^*∗∗*^	0.827^*∗∗∗*^	1.173^*∗∗∗*^	1.286^*∗∗∗*^	−2.227^*∗∗*^	−1.793^*∗∗*^	2.470^*∗∗∗*^	−0.464
	(0.201)	(0.198)	(0.318)	(0.329)	(0.339)	(0.363)	(0.906)	(0.719)	(0.516)	(1.084)
lninf	0.283^*∗∗∗*^	0.289^*∗∗∗*^	0.313^*∗∗∗*^	0.323^*∗∗∗*^	0.266^*∗∗∗*^	0.350^*∗∗∗*^	0.068	0.042	0.355^*∗∗∗*^	0.352^*∗∗*^
	(0.038)	(0.038)	(0.036)	(0.037)	(0.053)	(0.056)	(0.067)	(0.058)	(0.120)	(0.172)
*R * ^2^	0.656	0.652	0.767	0.744	0.802	0.773				
AR(1)							*p* < 0.001	*p* < 0.001	*p* < 0.001	*p* < 0.001
AR(2)							*p*=0.038	*p*=0.149	*p*=0.114	*p*=0.237
Hansen							*p*=0.708	*p*=0.664	*p*=0.568	*p*=0.517
Obs	510	510	510	510	510	510	480	480	480	480

Standard errors are reported in parentheses. ^*∗∗∗*^, ^*∗∗*^, and ^*∗*^ represent significance at 1%, 5%, and 10% levels, respectively. Symbol L. means a lag of one period (similarly hereinafter).

The article "Identifying the Impact of Industrial Agglomeration on China's Carbon Emissions Based on the Spatial Econometric Analysis" was published in 2023. Journal: J Environ Public Health.

**Table 4:** Moran's I statistical values of carbon emissions in 30 provinces of China from 2003 to 2019.

Year	*W1*			*W2*			*W3*		
	Moran's I	Z-stat	*p* value	Moran's I	Z-stat	*p* value	Moran's I	Z-stat	*p* value
2003	0.336^*∗∗∗*^	3.017	*p*=0.001	0.111^*∗*^	1.631	0.051	0.137^*∗∗∗*^	3.193	*p*=0.001
2004	0.381^*∗∗∗*^	3.369	*p* < 0.001	0.112^*∗*^	1.636	0.051	0.149^*∗∗∗*^	3.393	*p* < 0.000
2005	0.380^*∗∗∗*^	3.352	*p* < 0.001	0.098^*∗*^	1.480	0.069	0.144^*∗∗∗*^	3.303	*p* < 0.000
2006	0.377^*∗∗∗*^	3.334	*p* < 0.001	0.114^*∗∗*^	1.655	0.049	0.156^*∗∗∗*^	3.525	*p* < 0.000
2007	0.389^*∗∗∗*^	3.435	*p* < 0.001	0.121^*∗∗*^	1.744	0.041	0.162^*∗∗∗*^	3.639	*p* < 0.000
2008	0.403^*∗∗∗*^	3.564	*p* < 0.001	0.140^*∗∗*^	1.965	0.025	0.174^*∗∗∗*^	3.881	*p* < 0.000
2009	0.403^*∗∗∗*^	3.584	*p* < 0.001	0.143^*∗∗*^	1.998	0.023	0.173^*∗∗∗*^	3.882	*p* < 0.000
2010	0.422^*∗∗∗*^	3.745	*p* < 0.001	0.118^*∗∗*^	1.722	0.043	0.152^*∗∗∗*^	3.502	*p* < 0.000
2011	0.402^*∗∗∗*^	3.615	*p* < 0.001	0.102^*∗*^	1.556	0.060	0.132^*∗∗∗*^	3.155	*p*=0.001
2012	0.396^*∗∗∗*^	3.548	*p* < 0.001	0.131^*∗∗*^	1.880	0.030	0.145^*∗∗∗*^	3.387	*p* < 0.000
2013	0.376^*∗∗∗*^	3.379	*p* < 0.001	0.127^*∗∗*^	1.834	0.033	0.141^*∗∗∗*^	3.303	*p* < 0.000
2014	0.380^*∗∗∗*^	3.417	*p* < 0.001	0.134^*∗∗*^	1.911	0.028	0.142^*∗∗∗*^	3.325	*p* < 0.000
2015	0.352^*∗∗∗*^	3.192	*p* < 0.001	0.120^*∗∗*^	1.761	0.039	0.128^*∗∗∗*^	3.061	*p*=0.001
2016	0.321^*∗∗∗*^	2.923	*p*=0.002	0.119^*∗∗*^	1.744	0.041	0.125^*∗∗∗*^	2.990	*p*=0.001
2017	0.297^*∗∗∗*^	2.741	*p*=0.003	0.103^*∗*^	1.567	0.059	0.111^*∗∗∗*^	2.750	*p*=0.003
2018	0.330^*∗∗∗*^	3.034	*p*=0.001	0.137^*∗∗*^	1.966	0.025	0.136^*∗∗∗*^	3.229	*p*=0.001
2019	0.332^*∗∗∗*^	3.047	*p*=0.001	0.141^*∗∗*^	2.008	0.022	0.133^*∗∗∗*^	3.192	*p*=0.001

^*∗∗∗*^, ^*∗∗*^, ^*∗*^ represent significance at 1%, 5%, and 10% levels, respectively.

The article "Identifying the Impact of Industrial Agglomeration on China's Carbon Emissions Based on the Spatial Econometric Analysis" was published in 2023. Journal: J Environ Public Health.

**Table 5:** Spatial panel econometric results of the influence of SA and DA on carbon emissions.

Variable	*W1*		*W2*		*W3*	
	(1)	(2)	(3)	(4)	(5)	(6)
L.lnCE	0.969^*∗∗∗*^	1.022^*∗∗∗*^	0.965^*∗∗∗*^	0.999^*∗∗∗*^	0.973^*∗∗∗*^	0.989^*∗∗∗*^
	(0.022)	(0.021)	(0.023)	(0.021)	(0.023)	(0.021)
W × L.lnCE	−0.231^*∗∗∗*^	−0.192^*∗∗∗*^	−0.263^*∗∗∗*^	−0.273^*∗∗∗*^	−0.350^*∗∗*^	−0.309^*∗∗*^
	(0.068)	(0.069)	(0.089)	(0.089)	(0.150)	(0.149)
W × lnCE	0.287^*∗∗∗*^	0.305^*∗∗∗*^	0.356^*∗∗∗*^	0.396^*∗∗∗*^	0.558^*∗∗∗*^	0.672^*∗∗∗*^
	(0.062)	(0.062)	(0.084)	(0.082)	(0.141)	(0.135)
lnSA	0.091^*∗∗∗*^		0.087^*∗∗*^		0.065*∗*	
	(0.040)		(0.037)		(0.038)	
lnDA		−0.013^*∗*^		−0.020^*∗∗∗*^		−0.018^*∗∗*^
		(0.008)		(0.007)		(0.007)
lnpgdp	0.004	0.008	0.004	0.014	−0.005	−0.004
	(0.031)	(0.032)	(0.031)	(0.032)	(0.032)	(0.032)
lner	0.054^*∗∗*^	0.054^*∗∗*^	0.048^*∗∗*^	0.041^*∗∗*^	0.049^*∗∗*^	0.043^*∗∗*^
	(0.021)	(0.021)	(0.021)	(0.021)	(0.021)	(0.021)
[lner]^2^	−0.006^*∗∗*^	−0.007^*∗∗*^	−0.006^*∗∗*^	−0.005	−0.006^*∗*^	−0.005
	(0.003)	(0.003)	(0.003)	(0.003)	(0.003)	(0.003)
ur	−0.428^*∗∗∗*^	−0.552^*∗∗∗*^	−0.395^*∗∗∗*^	−0.466^*∗∗∗*^	−0.386^*∗∗*^	−0.409^*∗∗∗*^
	(0.148)	(0.150)	(0.150)	(0.151)	(0.150)	(0.151)
lninf	−0.087^*∗∗∗*^	−0.116^*∗∗∗*^	−0.077^*∗∗∗*^	−0.088^*∗∗∗*^	−0.079^*∗∗∗*^	−0.090^*∗∗∗*^
	(0.023)	(0.024)	(0.023)	(0.023)	(0.023)	(0.023)
Log-likelihood	875.111	860.107	877.054	870.349	876.962	870.310
Obs	510	510	510	510	510	510

Standard errors are reported in parentheses. ^*∗∗∗*^, ^*∗∗*^, and ^*∗*^ represent significance at 1%, 5%, and 10% levels, respectively.

**Table 6:** Estimation results of the effects of SA and DA on carbon emissions for the subsample with W1.

Variable	*Eastern region*		*Central region*		*Western region*	
	(1)	(2)	(3)	(4)	(5)	(6)
L.lnCE	1.192^*∗∗∗*^	1.195^*∗∗∗*^	1.599^*∗∗∗*^	1.581^*∗∗∗*^	0.928^*∗∗∗*^	0.908^*∗∗∗*^
	(0.047)	(0.043)	(0.097)	(0.097)	(0.041)	(0.042)
W × L.lnCE	−0.102	−0.071	1.803^*∗∗∗*^	1.706^*∗∗∗*^	0.049	0.036
	(0.089)	(0.090)	(0.238)	(0.231)	(0.147)	(0.145)
W × lnCE	0.240^*∗∗∗*^	0.280^*∗∗∗*^	0.171	0.174	0.364^*∗∗∗*^	0.350^*∗∗∗*^
	(0.080)	(0.081)	(0.148)	(0.151)	(0.108)	(0.108)
lnSA	0.003		0.211^*∗*^		0.208^*∗∗∗*^	
	(0.065)		(0.113)		(0.078)	
lnDA		−0.016		−0.007		−0.043^*∗∗∗*^
		(0.014)		(0.014)		(0.015)
lnpgdp	−0.226^*∗∗∗*^	−0.225^*∗∗∗*^	−0.800^*∗∗∗*^	−0.772^*∗∗∗*^	0.367^*∗∗∗*^	0.354^*∗∗∗*^
	(0.055)	(0.055)	(0.127)	(0.127)	(0.089)	(0.088)
lner	0.011	0.018	0.113	0.077	0.099^*∗∗*^	0.100^*∗∗*^
	(0.026)	(0.026)	(0.078)	(0.079)	(0.045)	(0.045)
[lner]^2^	0.000	−0.001	−0.015	−0.010	−0.015^*∗∗*^	−0.016^*∗∗*^
	(0.004)	(0.004)	(0.013)	(0.013)	(0.006)	(0.006)
ur	−0.474^*∗∗∗*^	−0.423^*∗∗*^	−2.713^*∗∗∗*^	−2.912^*∗∗∗*^	−2.628^*∗∗∗*^	−2.714^*∗∗∗*^
	(0.175)	(0.174)	(0.954)	(0.969)	(0.638)	(0.636)
lninf	−0.291^*∗∗∗*^	−0.315^*∗∗∗*^	0.062	0.051	−0.066	−0.068
	(0.039)	(0.040)	(0.098)	(0.098)	(0.042)	(0.042)
Log-likelihood	370.953	364.938	111.351	113.052	292.829	294.666
Obs	221	221	102	102	187	187

Standard errors are reported in parentheses. ^*∗∗∗*^, ^*∗∗*^, and ^*∗*^ represent significance at 1%, 5%, and 10% levels, respectively. The eastern region contains the following provinces: Zhejiang, Jiangsu, Beijing, Shanghai, Heilongjiang, Tianjin, Fujian, Hebei, Shandong, Guangdong, Hainan, Liaoning, and Jilin; the central region contains the following provinces: Jiangxi, Shanxi, Henan, Anhui, Hunan, and Hubei; the western region contains the following provinces: Ningxia, Chongqing, Inner Mongolia, Sichuan, Guangxi, Guizhou, Shaanxi, Yunnan, Qinghai, Xinjiang, and Gansu.

The article "Identifying the Impact of Industrial Agglomeration on China's Carbon Emissions Based on the Spatial Econometric Analysis" was published in 2023. Journal: J Environ Public Health.

**Table 7:** Robustness test results of the impact of SA and DA on carbon emissions.

Variable	*Adjusting the period*		*Remeasuring the variable*		*Economic weight matrix*	
	(1)	(2)	(3)	(4)	(5)	(6)
L.lnCE	0.951^*∗∗∗*^	1.009^*∗∗∗*^	0.956^*∗∗∗*^	0.985^*∗∗∗*^	0.968^*∗∗∗*^	1.007^*∗∗∗*^
	(0.025)	(0.024)	(0.021)	(0.020)	(0.023)	(0.021)
W×L.lnCE	−0.296^*∗∗∗*^	−0.264^*∗∗∗*^	−0.174^*∗∗*^	−0.160^*∗∗*^	−0.264^*∗∗∗*^	−0.273^*∗∗∗*^
	(0.072)	(0.073)	(0.073)	(0.073)	(0.098)	(0.099)
W×lnCE	0.308^*∗∗∗*^	0.321^*∗∗∗*^	0.259^*∗∗∗*^	0.273^*∗∗∗*^	0.361^*∗∗∗*^	0.394^*∗∗∗*^
	(0.066)	(0.067)	(0.063)	(0.063)	(0.090)	(0.089)
lnSA	0.136^*∗∗∗*^		0.088^*∗∗*^		0.096^*∗∗∗*^	
	(0.046)		(0.034)		(0.037)	
lnDA		−0.016^*∗*^		−0.016^*∗∗*^		−0.021^*∗∗∗*^
		(0.009)		(0.007)		(0.007)
lnpgdp	−0.002	0.004	−0.058^*∗*^	−0.012	0.007	0.020
	(0.037)	(0.039)	(0.033)	(0.032)	(0.032)	(0.032)
lner	0.045^*∗*^	0.042^*∗*^	0.038^*∗∗*^	0.035^*∗*^	0.046^*∗∗*^	0.039^*∗*^
	(0.024)	(0.025)	(0.019)	(0.019)	(0.021)	(0.021)
[lner]^2^	−0.004	−0.004	−0.005	−0.005	−0.006^*∗*^	−0.005
	(0.004)	(0.004)	(0.003)	(0.003)	(0.003)	(0.003)
ur	−0.311	−0.439^*∗*^	−0.077	−0.125	−0.426^*∗∗∗*^	−0.515^*∗∗∗*^
	(0.192)	(0.199)	(0.135)	(0.137)	(0.149)	(0.150)
lninf	−0.107^*∗∗∗*^	−0.124^*∗∗∗*^	−0.063^*∗∗∗*^	−0.071^*∗∗∗*^	−0.075^*∗∗∗*^	−0.086^*∗∗∗*^
	(0.029)	(0.030)	(0.021)	(0.021)	(0.023)	(0.023)
Log-likelihood	777.076	764.061	917.570	909.683	875.792	867.675
Obs	450	450	510	510	510	510

Standard errors are reported in parentheses. ^*∗∗∗*^, ^*∗∗*^, and ^*∗*^ represent significance at 1%, 5%, and 10% levels, respectively.

The article "Identifying the Impact of Industrial Agglomeration on China's Carbon Emissions Based on the Spatial Econometric Analysis" was published in 2023. Journal: J Environ Public Health.

## Data Availability

The experimental data used to support the findings of this study are available from the corresponding author upon request.
